# Correlation between Carotid Stenosis Degree and Blood Pressure Variability in Patients with Carotid Stenosis

This article has been retracted.

**DOI:** 10.1155/2022/4305015

**Published:** 2022-05-21

**Authors:** Junli Nie, Liang Hou, Baozhen Tan

**Affiliations:** Department of Cardiology, General Hospital of the Yangtze River Shipping, China

## Abstract

**Background:**

Carotid artery stenosis is one of the most serious diseases that endanger human health in contemporary times. It is a frequently occurring and common disease of the middle-aged and elderly people. Its incidence is increasing year by year, bringing a heavy economic burden to society and families. Whether there is a relationship between the degree of carotid artery stenosis and blood pressure variability is less studied.

**Aims:**

To investigate the correlation between the degree of carotid stenosis and blood pressure variability in patients with carotid stenosis.

**Materials and Methods:**

A total of 200 patients with carotid artery stenosis who were treated in our hospital from January 2017 to January 2020 were selected as the subjects of prospective study and were divided into mild stenosis according to the degree of carotid stenosis (carotid artery stenosis rate was 0-50%), moderate stenosis (carotid artery stenosis rate was between 50% and 70%), severe stenosis (carotid artery stenosis rate≧70%), and the control group with 50 cases each. The correlations between the hemodynamics, the degree of carotid artery stenosis, and blood pressure variability in patients with carotid artery stenosis were analyzed.

**Results:**

The levels of 24hSSD, 24hDSD, dSSD, dDSD, and nSSD in the mild stenosis group and moderate stenosis group were significantly higher than those in the control group. In the stenosis group, the levels of 24hSSD, 24hDSD, dSSD, dDSD, and nSSD in the severe stenosis group were significantly higher than those in the moderate stenosis group, with statistical significance (*P* < 0.05). The levels of PSV, EDV, and MV in the mild stenosis group and moderate stenosis group were lower than those in the control group, while the PI and RI indexes were higher than those in the control group. PI and RI levels were significantly higher than those in the mild stenosis group and moderate stenosis group (*P* < 0.05). Logistic analysis showed that EDV (*P* = 0.001, OR = 2.245, 95%CI = 1.638 ~ 3.078), SSD (*P* = 0.014, OR = 0.725, 95%CI = 0.528 ~ 0.996), and PSV (*P* = 0.001, OR = 1.970, 95%CI = 1.300 ~ 2.990) were closely related to the degree of carotid artery stenosis.

**Conclusion:**

Hemodynamics and blood pressure variability are related to the severity of carotid stenosis, which provides a reference and basis for clinical treatment of carotid stenosis.

## 1. Introduction

The causes of high blood pressure are not single, but mainly include related to tiny chemical assembly instructions inside of living thing factors, dietary nutrients, related to how people think and treat each other, stress, kidney-related factors, and neuroendocrine factors [1, 2]. There are many associations between higher blood pressure and neck artery narrowing, which is involved in crime in the how a disease started of dangerous blood vessel disease [3]. The creation and group of objects of dangerous blood vessel disease is ruled over by high blood pressure [4]. Due to the sudden increase of fluid pressure in the blood tube in the body, a swirl is created at its division into two positions, and the fluid flow in the blood tube in the body produces different stresses on the tube wall, which are usually divided into three types: fluid shear stress, axial stress, and press or force into a smaller space stress. The fluid shear stress is the most important [5, 6]. This study focused on exploring the relationship between the degree of neck artery narrowing of a passageway and blood pressure quality of changing over time or at different places, and the current research results are reported as follows.

## 2. Material and Methods

### 2.1. Research Object

Before enrollment, all patients in this study were given informed consent and signed the informed consent form. 200 patients with carotid artery stenosis who were treated in our hospital from January 2017 to January 2020 were selected as prospective study subjects. The degree of stenosis was divided into mild stenosis, moderate stenosis, and severe stenosis in 50 cases each. At the same time, 50 healthy subjects without carotid artery stenosis who were matched with baseline data such as age, gender, and occupation were selected as the control group.

### 2.2. Inclusion and Exclusion Criteria

Inclusion criteria are as follows: (i) all patients with carotid artery stenosis in this study met the diagnostic criteria for carotid artery stenosis in the “Chinese Guidelines for the Prevention and Treatment of Hypertension (Revised 2018)” [7]; (ii) the selected patients were conscious and able to express their wishes; and (iii) local sexual neurological symptoms and signs disappeared completely within 24 hours, and the number of episodes was small and the symptoms were the same each time.

## 3. Methods

### 3.1. Carotid Ultrasonography

All patients underwent carotid ultrasonography with X300 color Doppler ultrasound diagnostic apparatus (Siemens, Germany) within 7 days of hospitalization. Linear array probes with frequencies of 5 to 10 MHz were used. During the operation, the patient is in a supine position, and the head is tilted backward to fully expose the neck. The common carotid artery is detected in the order of the submandibular angle, the upper end of the clavicle, the posterior occipital angle, and the anterior border of the sternocleidomastoid muscle. Vessel diameter (D), peak systolic blood flow (PS), and peak diastolic blood flow (PD) were measured. Two-dimensional and color blood flow images (EDV), mean blood flow velocity (MV), resistance index (RI), pulsatility index (PI), etc. were used to determine the plaque situation. Blood flow status, carotid intima-media thickness (IMT), internal diameter of common carotid artery, presence or absence of plaque, plaque location, size, shape, echo, and spectral shape were observed.

### 3.2. All-Weather Ambulatory Blood Pressure Monitoring

Within 3 days of admission, all patients were monitored with AB-PM6100 noninvasive portable ambulatory blood pressure monitor (Welch Allyn, USA). During the day (6:00-2:00), monitoring was performed once for 30 minutes and at night (once at 22:00 at 6:00 a day) with an interval of 1 hour. The measured data were input into the computer for processing, and the monitoring indicators were 24 h systolic blood pressure (24hSSD), 24 h diastolic blood pressure (24hDSD), daytime systolic blood pressure (dSSD), daytime diastolic blood pressure (dDSD), nighttime diastolic blood pressure (nSSD), and nocturnal diastolic blood pressure (nSSD).

## 4. Observation Indicators

### 4.1. Carotid Artery Stenosis Grading

Internal carotid artery stenosis rate = (the original inner diameter of the plaque at the plaque site − the current inner diameter)/the original inner diameter × 100%.

### 4.2. Variability Index of Hypertension

Blood pressure rhythm changes are expressed by nighttime blood pressure drop rate: nocturnal blood pressure drop rate = [(daytime average blood pressure − nighttime average blood pressure)/daytime average blood pressure] × 100%. According to the different speeds of blood pressure drop at night, the change of blood pressure circadian rhythm is divided into 4 types, namely, dipper (nocturnal blood pressure drop rate of 10%~20%), nondipper (nocturnal blood pressure drop rate < 10%), reverse-dipper type (nocturnal blood pressure rise rate > 20%), and super-dipper type (nocturnal blood pressure fall rate > 20%); they are mainly systolic blood pressure. The carotid artery flow is the blood flow per unit area of the bilateral intracranial arteries. The sum of the flow: the cerebral artery flow is the sum of the blood flow of the bilateral intracranial arteries and the bilateral vertebral arteries.

## 5. Statistical Analysis

All statistical data in this study were entered into Excel software by the first author and the corresponding author, respectively, and the statistical processing software was SPSS25.0 for calculation. Count data expressed as a percentage (%) were tested by *χ*^2^. Univariate and logistic multivariate regression analysis was used to compare the influencing factors, and the risk factors with significant differences were screened. The statistical significance was *P* < 0.05.

## 6. Results

### 6.1. General Data Comparison

There were no a big change in numbers that means something important differences in the general data such as female status, average age, average course of disease, how fat or skinny you are based on height and weight, and case type between the two groups of patients (*P* > 0.05). See Table 1.

### 6.2. Blood Pressure Detection Indicators

The levels of 24hSSD, 24hDSD, dSSD, dDSD, and nSSD in the mild stenosis group and moderate stenosis group were significantly higher than those in the control group. The detection index levels were significantly higher than those in the moderate stenosis group, with statistical significance (*P* < 0.05). See Figure 1.

### 6.3. Hemodynamic Comparison

The levels of PSV, EDV, and MV in the mild stenosis group and moderate stenosis group were lower than those in the control group, while the PI and RI indexes were higher than those in the control group. PI and RI levels were significantly higher than those in the mild stenosis group and moderate stenosis group (*P* < 0.05). See Figure 2.

### 6.4. Logistic Multivariate Analysis

Assign the variables with significant differences tested in the above table, namely, EDV (normal = 1, abnormal = 2), SSD (normal = 1, abnormal = 2), PI (normal = 1, abnormal = 2), RI (normal = 1, abnormal = 2), and PSV (normal = 1, abnormal = 2). Logistic analysis showed that EDV (OR = 2.245, 95%CI = 1.638 ~ 3.078), SSD (OR = 0.725, 95%CI = 0.528 ~ 0.996), and PSV (OR = 1.970, 95%CI = 1.300 ~ 2.990) were significantly different from each other. The degree of carotid stenosis is closely related. See Table 2.

## 7. Sleep Quality Score Comparison

Before nursing, there was no significant difference in sleep quality scores between the two groups of breast cancer patients with liver metastases (*P* > 0.05). After nursing, the sleep quality scores, increased awakening scores, sleep instability scores, and night terrors scores of breast cancer patients with liver metastases in the two groups were significantly improved, and the sleep quality scores of the observation group were significantly lower than those of the comparison group. There was statistical significance (*P* < 0.05). See Figure 3.

## 8. Mental State Comparison

Before nursing, there was no significant difference in the psychological state scores between the two groups of breast cancer patients with liver metastases (*P* > 0.05). After nursing, the anxiety score, depression score, fatigue and distress score, and anger score of the two groups of breast cancer patients with liver metastases were significantly improved, and the psychological state score of the observation group was significantly lower than that of the comparison group, and statistics showed that the difference was statistically significant (*P* < 0.05). See Figure 4.

## 9. Self-Care Ability Score Comparison

There was no significant difference in the scores of self-care ability of the two groups before nursing (*P* > 0.05). After nursing, the scores of self-care skills, self-responsibility, health knowledge, and self-concept of the observation group were higher than those of the comparison group. The statistical difference was shown to be statistically significant (*P* < 0.05). See Figure 5.

## 10. Quality of Life Score Comparison

There was no significant difference in the quality of life scores between the two groups before nursing (*P* > 0.05). After nursing, the scores of mental vitality, social interaction, emotional limitation, and mental status of the observation group were significantly higher than those of the comparison group, and the difference was statistically significant (*P* < 0.05). See Figure 6.

## 11. Discussion

Another important mechanism is autonomic regulation, which mainly affects long-term blood pressure variability [8]. In addition, the central nervous system, humoral-endocrine function, spirit, environment, physical activity, and vasomotor activity of vascular smooth muscle also have certain regulatory effects on blood pressure variability [9]. In addition to congenital factors, scholars generally believe that carotid artery stenosis is consistent with the pathogenesis of atherosclerosis, and the formation of atherosclerosis is dominated by hypertension [10, 11]. The fluid flowing in the blood vessel produces different stresses on the tube wall, which are generally divided into fluid shear stress, axial stress, and compressive stress, among which the fluid shear stress is the most important [12].

This study investigated the correlation between the degree of carotid stenosis and blood pressure variability in patients with carotid stenosis. The results showed that the levels of 24hSSD, 24hDSD, dSSD, dDSD, and nSSD in the mild stenosis group and moderate stenosis group were significantly higher than those in the control group. The 24hSSD, 24hDSD, dSSD, dDSD, and nSSD index levels in the stenosis group and severe stenosis group were significantly higher than those in the mild stenosis group. It can be seen that with the increase of the degree of carotid stenosis, the blood flow velocity gradually decreases, while the peripheral resistance increases significantly. The reason is that the wall thrombus and atherosclerotic plaques at the sclerotic stenosis of the arteries cause microthrombus embolism, which slows down the blood flow and increases the peripheral resistance [13].

Logistic analysis showed that EDV, SSD, and PSV were closely related to the degree of carotid artery stenosis. The mechanism may be that the large fluctuation of blood pressure for a long time will increase the shear force on the inner wall of the blood vessel, thereby aggravating the damage to the vascular endothelium, resulting in an increase in blood flow resistance and a decrease in vascular compliance [14]. It further accelerates the occurrence and development of atherosclerosis and then promotes carotid artery stenosis to form mouth force [15]. Therefore, hypertension (fluctuating blood pressure) affects the morphology, structure, and function of vascular endothelial cells, as well as vascular permeability [16]. It shows that the change of blood pressure circadian rhythm is related to carotid artery stenosis. The mechanism may be that blood pressure in patients with nondipper rhythm has insufficient nocturnal blood pressure drop, resulting in the disappearance of normal circadian fluctuations [18]. As a result, the nighttime blood pressure is kept at a high level for a long time, resulting in a high load state of the vascular system for a long time, and the long-term high load of the blood vessels will reduce the elasticity of the arterial wall and the vascular compliance [19]. Thereby increasing vascular resistance, resulting in a decrease in blood flow velocity and shear stress, thereby promoting the formation of atherosclerosis and carotid artery stenosis [20]. Studies have shown that the blood pressure variability of healthy people is the smallest, and their 24-hour blood pressure is a dipper rhythm; that is, the nighttime blood pressure is 10% lower than the daytime blood pressure [21–23]. In recent years, many studies have shown that abnormal blood pressure circadian rhythm is closely related to the occurrence and development of atherosclerosis [24]. The structure of the carotid arteries can regulate the contraction and relaxation of blood vessels, and the physiological changes of the vessel wall can be balanced under long-term slow mechanical stimulation [25]. Although most of the hypertensive patients in China have received antihypertensive treatment, the antihypertensive treatment is not always under the guidance of doctors, and the antihypertensive treatment is not continuous [26]. The blood pressure of these patients is often in arrhythmic changes, so the incidence of arterial stenosis is higher [27]. In addition, the stress fibers of endothelial cells cultured under static conditions have no directional arrangement, and after applying shear stress after 72 hours, the stress fiber arrangement is consistent with the flow field [28]. After 72 hours of shear stress, the stress fibers were rearranged, and the morphology of endothelial cells also changed, from round to long spindle, consistent with the direction of blood flow shear stress [29]. Multivariate logistic analysis showed that EDV, SSD, and PSV were the influencing factors of carotid artery stenosis. Studies have shown that the incidence of hypertension in patients with carotid artery stenosis is significantly higher than the general population [30].

Like other body structure-related limits/guidelines of the body, blood pressure is not static. In common and regular people and most high blood pressure-related patients, blood pressure will go up and down with changes in sleep and wakefulness, day and night, rest and activity, and body position. This blood pressure quality of changing over time or at different places, which is the body's neuroendocrine energetic/changing regulation, results in a complete and thorough balance [31]. Since blood pressure quality of changing over time or at different places was recognized in the 1980s, it has received more attention over the last few years. As an important indicator to watch obey blood pressure ups and downs, blood pressure quality of changing over time or at different places has been used in medicine-based and scientific research [32]. Generally, the mean standard moving away of blood pressure watching/supervising reflects the importance of different versions, and blood pressure quality of changing over time or at different places is closely related to arterial elastic function and the degree of dangerous blood vessel disease [33]. A study of carotid intima thickness in high blood pressure-related patients found that not only 24 h systolic blood pressure levels but also blood pressure ups and downs were related to related to what holds something together and makes it strong changes in large blood vessels from the busy roads [34]. Common neck artery intima-media thickness and the standard moving away or coefficient of different versions of 24 h systolic blood pressure and pulse pressure were significantly positively related, and the relationship remained after multivariate moving backward analysis. Carotid dangerous blood vessel disease is related to blood pressure quality of changing over time or at different places [35]. Studies have shown that the development or increase over series of events or things of carotid intima-media thickness increases by 0.005-0.012 mm/year for every 1 mmHg increase in blood pressure quality of changing over time or at different places expressed by standard moving away, and with the increase of daytime systolic blood pressure quality of changing over time or at different places, the number of times something happens of early carotid dangerous blood vessel disease increases. The relative risk was increased a lot [36]. For early identification of a disease or problem, or its cause of dangerous blood vessel disease, the unsteadiness of daily blood pressure in common and regular people in the early stage is mostly 10% lower than that in the daytime, showing dipper blood pressure with “double peaks and one valley” or “double peaks and double valleys” [37]. High blood pressure-related patients are mostly having dipper-type blood pressure, and some are nondipper-type and super-dipper-type, and some even have made higher blood pressure at night (reverse-dipper-type) [38]. Changes in the common and regular daily rhythm of blood pressure are not only the result of a too much of one thing and not enough of another in the blood vessel-related law-based machine after sudden and serious stroke but also a high-risk factor for intelligent/brain-based infarction [39]. Studies have shown that the number of times something happens of different from what is usually expected daily rhythm in the high blood pressure group with the heart, brain, and organ that creates urine damage is much higher than that in the high blood pressure group, and the target organ damage group is ruled over by nondipper rhythms. This study shows that carotid dangerous blood vessel disease is obvious and extreme in patients with different from what is usually expected daily rhythm [40]. Loss of blood pressure daily rhythm significantly worsens the degree of dangerous blood vessel disease. Changes in the daily rhythm of blood pressure can keep blood tubes in the body in a high load state, reduce arterial following the doing as you are told, increase blood vessel-related resistance, and reduce blood flow rate and shear stress, by that/in that way helping showing in a good way the creation and group of objects of dangerous blood vessel disease and damaging the structure and function of blood tubes in the body.

There are still some limits in this study. The research objects are few, and the multi-deadliness of old patients leads to too many confusing factors in the study, which affects the experimental results. There was no association between hyperdipper patients and carotid intima injury, and no comparison was made with nondipper and reverse-dipper patients to understand the association of nondipper and reverse-dipper patients with carotid intima injury. At the same time, the study did not track the subjects and did not find out whether the daily rhythm of blood pressure before and after act of letting someone speaking the truth about something bad was agreeing matching up working regularly with that during time in a hospital, allowing for better supervising of blood pressure ups and downs and changes in daily rhythms. When looking at blood pressure quality of changing over time or at different places between people, changes were found to be strongly connected with later risk of related to the heart and blood vessels events, with some studies suggesting that in patients with blood vessel-related disease, higher blood pressure quality of changing over time or at different places is related to a higher risk of related to the heart and blood vessels events higher.

## 12. Conclusion

In the end, hemodynamics and blood pressure quality of changing over time or at different places are related to the extreme harshness of carotid narrowing of a passageway, which provides a reference and basis for medicine-based treatment of carotid narrowing of a passageway.

## Figures and Tables

**Figure 1:** Comparison of blood pressure detection indicators between the two groups of patients. According to the test standard of *α* = 0.05, the blood pressure index levels of 24hSSD, 24hDSD, dSSD, dDSD, nSSD, and other blood pressure indicators of the 4 groups of patients were expressed as the mean ± SD and were analyzed by the repeated measures variance test. Mild stenosis group, moderate stenosis group. The levels of 24hSSD, 24hDSD, dSSD, dDSD, and nSSD were significantly higher than those in the control group, the blood pressure detection index levels in the moderate stenosis group and the severe stenosis group were significantly higher than those in the mild stenosis group, and the blood pressure detection index levels in the severe stenosis group were significantly higher than those in the moderate stenosis group (*P* < 0.05).

**Figure 2:** Comparison of hemodynamics between the two groups of patients. According to the test standard of *α* = 0.05, the levels of PSV, EDV, MV, and other hemodynamic indexes in the 4 groups were expressed as the mean ± SD and were analyzed by the repeated measures variance test. The levels of PSV, EDV, and MV in the mild stenosis group and moderate stenosis group were lower than those in the control group, while the PI and RI indexes were higher than those in the control group. PI and RI levels were higher than those in the mild stenosis group and moderate stenosis group (*P* < 0.05).

**Figure 3:** Comparison of sleep quality scores. According to the test standard of *α* = 0.05, the scores of sleep quality (a), increased arousal score (b), sleep instability score (c), and sleep disturbance scores of the two groups of breast cancer patients with liver metastases after nursing care and night terrors scores (d) were significantly improved, and the sleep quality score in the observation group was significantly lower than that in the comparison group. Values are expressed as the mean ± SD and analyzed by the independent sample *t*-test. After nursing, the observation group's sleep quality score, increased arousal score, sleep instability score, and night terrors score were lower than those of the comparison group (*P* < 0.05).

**Figure 4:** Comparison of mental state scores. According to the test standard of *α* = 0.05, the anxiety score (a), depression score (b), fatigue and distress score (c), and anger score (d) of the two groups of breast cancer patients with liver metastases after nursing were significantly improved, and the psychological state score of the observation group was significantly lower than that of the comparison group. Values are expressed as the mean ± SD and analyzed by the independent sample *t*-test. The anxiety score, depression score, fatigue and distress score, and anger score of the observation group after nursing were lower than those of the comparison group (*P* < 0.05).

**Figure 5:** Self-care ability score comparison. There was no significant difference in the scores of self-care ability between the two groups of patients before nursing (*P* > 0.05). Health knowledge score (c) and self-concept score (d) were significantly improved, and the observation group's self-care ability score was significantly higher than that of the comparison group. According to the test standard of *α* = 0.05, the values were expressed as the mean ± SD which indicates that, using independent sample *t*-test analysis, the nursing skill score, self-responsibility score, health knowledge score, and self-concept score of the observation group after nursing were higher than those of the comparison group (*P* < 0.05).

**Figure 6:** Comparison of quality of life scores. There was no significant difference in the quality of life scores between the two groups before nursing (*P* > 0.05). After nursing, the scores of mental vitality (a), social interaction (b), the emotional restriction score (c), and the mental status score (d) were significantly improved, and the self-protection ability score of the observation group was significantly higher than that of the comparison group. According to the test standard of *α* = 0.05, the value was expressed as the mean ± SD, and the independent samples *t*-test was used for analysis. After nursing, the observation group had higher scores of mental vitality, social interaction, emotional limitation, and mental status than the comparison group (*P* < 0.05).

**Table 1:** Comparison of general data of the two groups of patients (*n*, $\bar{x}\pm s$).

Group	Gender (men/women)	Average age (year)	Average disease duration (moon)	Body mass index (kg/m^2^)	Case type		
					Cerebral infarction	Headache	Other
Comparison group (50)	24/26	31.78 ± 4.32	11.34 ± 3.25	27.78 ± 2.32	22	16	12
Mild stenosis (50)	22/28	31.62 ± 4.66	11.31 ± 3.64	27.62 ± 2.66	18	22	10
Moderate stenosis (50)	23/27	33.34 ± 1.25	10.51 ± 2.32	32.78 ± 3.32	19	21	10
Severe stenosis (50)	21/29	34.76 ± 1.64	9.55 ± 2.11	33.62 ± 3.66	21	17	12
*χ* ^2^/*F*	0.169	0.169	0.025	0.020	0.327		
*P*	0.506	0.506	0.965	0.984	0.849		

**Table 2:** Logistic multivariate analysis.

	*β*	S.E.	Wald *χ*^2^	*P*	OR	95% CI
SSD	0.152	0.081	16.797	0.014	0.725	0.528~0.996
EDV	0.1149	0.161	25.236	0.001	2.245	1.638~3.078
PI	0.101	0.175	0.336	0.562	1.107	0.786~1.599
RI	0.267	0.165	2.606	0.106	1.305	0.945~1.1144
PSV	0.6114	0.119	19.450	0.001	1.970	1.300~2.990

## Data Availability

No data were used to support this study.
